# Molecular Characteristics and Prognostic Role of MFAP2 in Stomach Adenocarcinoma

**DOI:** 10.1155/2022/1417238

**Published:** 2022-03-21

**Authors:** Fenfen Tang, Chaoyi Hu, Zhi Long, Yanping Liu, Guoqing Li

**Affiliations:** Department of Gastroenterology, Second Affiliated Hospital, University of South China, Hengyang, China

## Abstract

Molecular characteristics and prognostic role of MFAP2 were by no means stated. The MFAP2 expression and prognostic prices in this study, with Cox analysis, was employed to develop a predictive fee for MFAP2. To know about coexpression and practical networks associated with MFAP2, LinkedOmics and GEPIA2 have been used. MFAP2 expression has been increased and verified in many unbiased coalitions in TCGA-STAD tumor tissues. In addition, in each TCGA and various cohorts, increased MFAP2 was linked with lower survival. Evaluation by Cox revealed the unbiased danger to average survival, disease-specific survival, and progression-free survival of STAD used to be due to the elevated expression of MFAP2. Active community assessed the MFAP2, through which more than a few cancer-associated kinases and E2F household pathways are regulated, which shows that MFAP2 affects RNA transportation, oocyte meiosis, spliceosome, and ribosome biogenesis. MFAP2 can predict and is linked to the prediction of STAD independently. The closure of the MFAP2 link to the macrophage marker genes is, in particular, the achievable core of immune response.

## 1. Introduction

Gastric adenocarcinoma (STAD) is the most common malignant tumor of the digestive tract. Despite the overall increase in the diagnosis and treatment of STAD in the past decades, the incidence rate and mortality of STAD are still increasing due to the lack of early diagnosis and active treatment [1]. If STAD patients are recognized and dealt with early on, either with endoscopy or with surgery, the price for five years must, nevertheless, be over 90%. Therefore, the real-time prediction of STAD greatly increases the estimated value. Therefore, it is necessary to identify new candidate genes that play a key role in initiating and improving STAD and help reduce mortality prices and improve prediction [2–4].

Thanks to the constant innovation from the applied sciences in microarray and high-performance sequencing, the health center, particularly in scientific oncology, has identified a wider variety of biomarkers and therapeutic targets [5]. The Cancer Genome Atlas (TCGA) is an extensive database that provides publicly available genetic and medical evidence for the majority of malignancies. With this database, researchers may study the biology and pathophysiology of cancer in-depth and accurately. In addition, TCGA helps to predict and personalize cancer by developing new candidate genes and scientific facts associated with the majority of malignancies. Coexpression assessment is a viable way to build networks of scale-free gene coexpression [6]. Weighted gene coexpression community assessment (WGCNA) has been widely used for the analysis of large-scale statistical units and modules of highly connected genes. Moreover, WGCNA has been used to check linkages between genetic units and science effectively and to develop feasible applicant biomarkers with several types of cancer, prostate, oesophageal, and most cancers of the cervix. WGCNA, therefore, offers a deliberate interpretive device for most cancer biology and introduces fresh insights into the molecular etiology and prognosis of cancer [7–9].

## 2. Methods

### 2.1. Differential Expression of MFAP2

TCGA-STAD gene expression statistics profiles for patients and the scientific data for patients, such as age, sex, tumor stage, TNM classification, and survival status, available for download through the TCGA portal (https://portal.gdc.cancer.gov/) (assignment ID: TCGA-STAD) were obtained.

The Wilcoxon test, combined with unpaired or paired testing, was used for the TCGA-STAD cohort, differential STAD mRNA in tumor, and healthy tissues. Oncomine is a microarray database of most cancers and a statistics mining platform primarily based on the web (version 4.5: https://www.oncomine.org/). Oncomine recognized MFAP2 in STAD or normal tissues for its degree of mRNA expression for reproductive diversity. The following screening factors were selected to determine the content to cover in this test on Oncomine: (1) “Type of an analysis” was set to “cancer and daily analysis” once, “cancer” type was established at “Stomach adenocarcinoma” once, (2) “Transparency” was set to “*p* value<; 0.05,” and “GENE RANK” was set to “ALL.” The most common transcriptome information online analyses for cancers are UALCAN (http://ualcan.path.uab.edu/) and based mostly on a majority of the public transcriptome cancer records (TCGA and MET500 transcriptome sequencing). The “CPTAC analysis” module of UALCAN allows for the use of validation/discovery datasets of the UALCAN protein expression assessment options. UALCAN identified the expression of MFAP2 protein between STAD and the average stomach.

### 2.2. Analysis of MFAP2 Survival

The survival assessment of MFAP2 in the TCGA-STAD cohort by the Kaplan–Meier evaluation and log-rank test was performed. Kaplan–Meier Plotter is the Internet biomarker assessment tool based mostly on meta-analysis for breast, ovarian, lung, gastric, and liver cancer. Kaplan–Meier is a website for biomarker assessment. Furthermore, the affiliation of MFAP2 to STAD patients has been studied with a forecast scan, and the Kaplan–Meier plotter. SurvMiner and the R Survival programs conducted TCGA-STAD assessment and prognostics scanning. For belly adenocarcinoma and GEPIA, an association between MFAP2 expression and DFS has been assessed; we are using the UALCAN database for OS MFAP2 expression.

### 2.3. Analysis and LinkedOmics

LinkedOmics (http://www.linkedomics.org) and GEPIA2 database are open network sites that include many omics data for all 32 cancer types of TCGA. We utilize Pearson to look at the statistical characteristics of MFAP2 coexpression in the LinkFinter module of LinkedOmics. The effects are shown as a volcano, warmth map, or scatter map. The gene-target enrichment, the kinase-target enrichment, the transcription-target enrichment were based on the gene-packet enhancement analysis and the LinkInternet Interpreter module LinkedOmics (LinkInterpreters) (GSEA). The grade was formerly based mainly on an error detection fee (FDR). GEPIA2 database (httpwwyepi2. Cancer-PKU.cn/) is an online service used to study RNA-sequencing data on the use of modern processing pipelines for the use of 9,736 tumors and 8,587 daily TCGA and GTEX samples. GEPIA2 was utilized to create the warmth survival map and survival curve of the critical kinase of the coexpressed genes.

## 3. Results

### 3.1. MFAP2 mRNA in STAD Samples Is Overexpressed

The utilization of the TCGA portal and FIREBROWSE was initially recognized when MFAP2 mRNA was expressed in normal tissues and malignant tissues. The effects revealed comparable daily tissues by the stage of MFAP2 expression in tumor tissue. In contrast, we purposefully expressed MFAP2 mRNA in STAD and surface tissues, which was noticeably more significant than the expression of MFAP2 mRNA in STAD's tissues than in daily tissues. Next, the UALCAN was once performed with a more outstanding specific and distinct MFAP2 mRNA expression evaluation in STAD. The results of the examination of subgroups based mainly on the nodal metastasis, the nature of most cancer stages, and the grade of tumors suggested that the MFAP2 mRNA grades of STAD patients were substantially higher than the corresponding group.  Figure 1 shows the MFAP2 mRNA in STAD samples.

### 3.2. The Clinical Features of STAD Patients Are Related with MFAP2 Expression

So far, there has been almost no research that states a link between MFAP2 expression and human STAD's scientific prognosis. Thus, the influence of the MFAP2 on the survival index was evaluated using a plotter tool from Kaplan–Meier, which confirmed that good regulation of expression of MFAP2 was once significantly associated with shorter FP and PPS. The UALCAN database also confirms that the OS has been shortened of those with elevated MFAP2 levels. We also found that patients with excessive levels of MFAP2 expression had shorter DFS from the GEPIA database.  Figure 2 shows the results of the survival analysis.

### 3.3. MFAP2 Enrichment Protein Interactions and Analysis

STRING was employed once to achieve the interplay between MFAP2 and several binding proteins. The consequences have shown that various proteins, such ELN, EFEMP2, and FBLN1 are expected to bind to MFAP2 immediately. Therefore, we have performed a GO and KEGG pathway analysis to detect the organic characteristics of these co-DEGs. The GO Annotation describes the major body strategies, mobile (nucleus), and molecular characteristics of MFAP2 (protein bind) biology (response to stimulation and herbal regulation).  Figure 3 shows the MFAP2 enrichment and protein interactions assessment.

## 4. Discussion

Our first research found that MFAP2 may be employed as a proto-oncogene of STAD and may be employed in the entire mining of public databases as a manageable biomarker. We have further investigated the differential coexpression of STAD and have shown its organizational significance in most cancer growth by identifying a feasible signage route for STAD. The datasets Oncomine, UALCAN, and GEPIA indicate that MFAP2 is expressed mainly in STAD. The survival assessment of Kaplan–Meier also revealed that patients with expanded MFAP2 levels had reduced OS and PPS. Furthermore, the MFAP2 amount of methylation is contradictory to protein expression, which shows a low level [10].

The STAD molecular pathways have not been fully implemented, despite ample experimental research. Most unrecognized people with early STAD are no longer suitable for healing, leading to a poor prognosis. It is critically required to use diagnostic and therapeutic markers. The evaluation of bioinformatics plays a critical role in most cancer research and increases the assessment of cancer using genomic information with systemic methods to bioinformatics. We have studied MFAP2 expression in belly adenocarcinoma (STAD) and many different types of cancer in humans in the present work. We found that more than a few cancers once had MFAP2 elevated. In contrast to the daily tissues linked with survival probability, OS, and DSS, we have found that MFAP2 was overexpressed in STAD. In addition, we conducted in vitro investigations that demonstrated that knuckling of MFAP2 suppressed the proliferation and migration of ductal adenocarcinoma cells, which might constitute a biomarker for STAD, to examine whether or not MFAP2 silencing is contributing to the suppression of tumors. Several evaluations of fibrillin-1 mutant and MAGP-1 (MFAP2)-deficient mice showed identical skeletal characteristics. MFAP2 and fiber line 1 overlap adjusts the variety of the osteoclast and the absorption of the bone. Research suggests that MFAP2 is not needed for elastic fiber meetings in mice but is required for various tissue homeostasis or distinguishment techniques [11–13]. Thus, these fibrillin mutations can also change the ability of fibrillin to bind to MFAP2, mainly the disease's onset and worsening. Previous investigations showed that versions, the vast extracellular proteoglycan matrix, were found in conjunction with fibrillin-1, which played a critical role in tumor invasion and metastasis. Our recent results show that MFAP2 suppression can increase in vitro migration and proliferation. Together, MFAP2 can enhance and develop STAD through its interaction with the mutant fibrillin-1. The future study must examine whether or not fibrillin-1 is linked to MFAP2 in STAD cells. Then, we found that the MFAP2 expression once was at the marvellous histologic stage. MFAP2 is highly expressed at the highest stage, where MFAP2 predominantly refers to the ideal length of STAD, which shows a possible association between MFAP2 expression and STAD disease symptoms. We thus carried out the TCGA-STAD survival assessment, which shows that increased expression in MFAP2 was linked with dreadful results, which were once checked in the many impartial cohorts. In addition, Cox's analyses showed that MFAP2 formerly constituted an unmistakable danger to STAD. Our outcomes, therefore, show that overexpression of the MFAP2 occurs in STAD and that similar medical checks are essential as a practical diagnostic and prognostic marker [14, 15].

## 5. Conclusion

In the enhancement of STAD, MFAP2 can also play an essential function. MFAP2 can therefore also be a valuable forecast marker and an excellent anticancer objective in STAD.

## Figures and Tables

**Figure 1:** In STAD samples, MFAP2 is overexpressed. (a) Expression of MFAP2 mRNA in human cancer from *GeneCards*. (b) Expression of MFAP2 mRNA in STAD. (c, d, and e) MFAP2 mRNA expression differences, depending on the condition of nodal metastasis, M stage of cancer, and grade of tumor expression of MFAP2.

**Figure 2:** The results of microfibril-related protein two (MFAP2) expressions on prognosis in patients with stomach adenocarcinomas (STADs). (a, b) First progression (FP) and postprogressional survival (PPS) time evaluation for Kaplan–Meier patients primarily based on MFAP2 expression. (c) UALCAN database affiliation of the MFAP2 term with the OS. (d) The GEPIA database is assessed for the association of MFAP2 expression with DFS.

**Figure 3:** MFAP2 enrichment and protein interactions assessment. (a) Community of interactions between MFAP2 and several proteins. (b) WebGestalt has been acknowledged for the most crucial molecular activities, organic processes, and components related to MFAP2 biology.

## Data Availability

The analyzed datasets generated during the present study are available from the corresponding author on reasonable request.
